# Early Prediction of Epilepsy after Encephalitis in Childhood Based on EEG and Clinical Features

**DOI:** 10.1155/2023/8862598

**Published:** 2023-07-13

**Authors:** Xiaojuan Sun, Jinhua Zhao, Chunyun Guo, Xiaoxiao Zhu

**Affiliations:** Department of Pediatrics, The Second Affiliated Hospital of Nantong University, Nantong First People's Hospital, Nantong, Jiangsu, China

## Abstract

**Objective:**

The present study was designed to establish and evaluate an early prediction model of epilepsy after encephalitis in childhood based on electroencephalogram (ECG) and clinical features.

**Methods:**

255 patients with encephalitis were randomly divided into training and verification sets and were divided into postencephalitic epilepsy (PE) and no postencephalitic epilepsy (no-PE) according to whether epilepsy occurred one year after discharge. Univariate and multivariate logistic regression analyses were used to screen the risk factors for PE. The identified risk factors were used to establish and verify a model.

**Results:**

This study included 255 patients with encephalitis, including 209 in the non-PE group and 46 in the PE group. Univariate and multiple logistic regression analysis showed that hemoglobin (OR = 0.968, 95% CI = 0.951–0.958), epilepsy frequency (OR = 0.968, 95% CI = 0.951–0.958), and ECG slow wave/fast wave frequency (S/F) in the occipital region were independent influencing factors for PE (*P* < 0.05).The prediction model is based on the above factors: −0.031 × hemoglobin −2.113 × epilepsy frequency + 7.836 × occipital region S/F + 1.595. In the training set and the validation set, the area under the ROC curve (AUC) of the model for the diagnosis of PE was 0.835 and 0.712, respectively.

**Conclusion:**

The peripheral blood hemoglobin, the number of epileptic seizures in the acute stage of encephalitis, and EEG slow wave/fast wave frequencies can be used as predictors of epilepsy after encephalitis.

## 1. Introduction

Central nervous system infectious diseases are one of the most common diseases of the nervous system in children, and infectious diseases of the central nervous system in which pathogens mainly invade the brain parenchyma are called encephalitis [1, 2]. Encephalitis caused by direct invasion of the brain parenchyma by pathogenic microorganisms includes encephalitis caused by infections such as viruses, bacteria, fungi, and parasites, while autoimmune encephalitis or limbic lobehalitis related to tumors and immunity refers to inflammation-like diseases of the brain parenchyma caused by other nonspecific factors [3, 4]. The clinical manifestations of encephalitis are diverse; seizures are one of the most common manifestations. If not controlled in time, seizures can not only aggravate the irreversible damage of the primary disease but also lead to multisystem damage, directly affecting the prognosis and quality of life of patients [5, 6]. Most patients with encephalitis with seizures can be completely controlled with the improvement of the primary disease after etiological treatment and general supportive treatment, while some patients have seizures after the cure of encephalitis, which develop into postencephalitis epilepsy and require long-term use of antiepileptic drugs to control [7, 8].

Recurrent seizures have a serious impact on the physical and mental health of children, such as developmental delay, decreased IQ, loss of learning and working ability, poor social adaptability, personality changes, depression, which also bring a heavy burden to the family and society [9]. Therefore, the early identification, diagnosis, and treatment of patients with epilepsy after encephalitis have important clinical significance for improving their prognosis and living standards. However, large-scale clinical studies of factors associated with the acute phase of epilepsy after encephalitis are lacking, and there are significant differences in existing findings due to differences in inclusion criteria and sample sizes [10, 11].

The electroencephalogram (EEG) is the most important auxiliary examination method for the diagnosis of epilepsy, which can be used to clarify the diagnosis of epilepsy, determine seizure type, and determine epilepsy syndrome [12, 13]. Quantitative EEG converts the time-varying brain wave signals on the ordinary EEG into digital signals with the frequency of EEG power and transforms the EEG into objective and quantifiable values [14, 15]. In the present study, we designed the establishment and evaluation of an early prediction model of epilepsy after encephalitis in childhood based on ECG slow wave/fast wave frequency and clinical features.

## 2. Patients and Methods

### 2.1. Patients and Ethical Statement

This was a single-center, retrospective study. From May 2019 to December 2021, 255 patients with encephalitis at The Second Affiliated Hospital of Nantong University were included in the present study. Inclusion criteria: (1) Age, 3–12 years old; (2) Being diagnosed as encephalitis; (3) Having epilepsy in the acute stage of encephalitis; (4) Follow-up for at least 1 year after discharge. Exclusion criteria: (1) Complicated with malignant tumor, chronic infectious diseases (HIV, HCV, HBV, *Mycobacterium tuberculosis*, etc.), heart disease, and autoimmune disease; (2) Severe liver and kidney dysfunction; (3) Past history of epilepsy; (4) Loss of connection or death during follow-up; (5) Incomplete clinical data; (6) Unsigned informed consent. In addition, this study was reviewed and approved by the local hospital ethics committee.

### 2.2. Diagnosis of Encephalitis and Data Extraction

The clinical diagnosis of patients with encephalitis as follows: (1) the patient has more than one of the four symptoms of epileptic seizure, mental disorder, nervous system defect, and consciousness disorder; (2) Head imaging showed brain damage, abnormal cerebrospinal fluid (white blood cell number > 10^7^/L, protein content >0.5 g/L, intracranial pressure>175 mm H_2_O), accompanied by fever and other infectious symptoms, and abnormal EEG, and the patient had more than two of the above symptoms; (3) Other neurological diseases such as tumor, metabolic brain disease, and autoimmune encephalitis were excluded. Moreover, collect electronic case files of all patients with encephalitis and extract their baseline clinical characteristics, including age, gender, white blood cell count (WBC), neutrophil to lymphocyte ratio (NLR), hemoglobin, albumin, globulin, fever, consciousness disorder, epilepsy type, epilepsy frequency, and magnetic resonance imaging (MRI) images.

### 2.3. Electroencephalogram and Data Analysis

All patients with epilepsy have an EEG test. The room is quiet during the tracing, and during the examination, keep awake, close your eyes, relax, and do induction tests such as opening your eyes and hyperventilation. EEG detection parameter settings: filter channel 0.5–30 HZ, time constant 0.3, paper feed speed 3 cm/s, gain 100 u V = l cm, scalp resistance of each electrode does not exceed 5000Q. After selecting monopolar lead tracing for 1 minute, when the EEG signal was stable, the EEG signal sampling without artifacts and representing EEG background activity was selected, and each patient took 8s as 1 sampling unit, and 10 sampling units were selected intermittently. The ratio of EEG slow wave/fast wave frequency (ECG s value) was calculated by fast Fourier transform: ECG s value = ((*δ* + *θ*)/(*α*1 + *α*2 + *β*1 + *β*2)). *δ* (1.0 – 3.9 HZ), *θ* (4.0 – 7.9 HZ), *α*1 (8.0 – 10.0 HZ), *α*2 (10.1 – 13.9 HZ), *β*1 (14.0 – 19.9 Hz), and *β*2(20.0 − 30.0 Hz).

### 2.4. Statistical Analysis

Data was recorded in an Excel table and was analyzed using SPSS25.0 (IBM, USA). Counting data is expressed as a percentage, while metering data is expressed as (mean ± standard deviation). We use chi square test to compare the difference in counting data between the two groups and the student's *t*-test to compare the difference in measuring data between the two groups. The variables that met the criteria in univariate analysis were introduced into multivariate stepwise logistic regression to construct a prediction model in the training set. Receiver operating characteristic (ROC) curves were constructed, and the area under the curve (AUC) was calculated to assess the performance of the model in the diagnosis of epilepsy patients with cognitive functions [16, 17]. *P* < 0.05 indicated significant difference.

## 3. Results

### 3.1. General Characteristics of Patients with Encephalitis

A total of 255 patients with encephalitis were included in the present study, and they were randomly assigned to training and verification sets, 184 in training set and 71 in the verification set. We compared the baseline characteristics of encephalitis patients between the training set and validation set and found that there was no significant difference between these two groups, including age, gender, WBC, NLR, hemoglobin, albumin, globulin, fever, consciousness disorder, partial seizure, epilepsy frequency, intracranial inflammation by MRI, and electroencephalogram slow wave/fast wave frequency (*P* > 0.05) (Table 1).

### 3.2. General Characteristics of Encephalitis Patients with or without Postencephalitic Epilepsy

Of the 255 children with encephalitis included in the study, 46 patients had epilepsy one year after discharge (PE group), and 209 patients had no epilepsy (no-PE group). We compared the baseline characteristics of patients in the PE group and no PE group, including age, gender, WBC, NLR, hemoglobin, albumin, globulin, fever, consciousness disorder, partial seizure, epilepsy frequency, intracranial inflammation by MRI and electroencephalogram slow wave/fast wave frequency. We found that there was no significant difference between age, gender, WBC, NLR, albumin, globulin, consciousness disorder, partial seizure, and intracranial inflammation by MRI (*P* > 0.05), while the level of hemoglobin in the PE group were significantly lower than that in the no-PE group (*P* < 0.05), and the proportion of patients with fever, the proportion of patients with epilepsy frequency ≥10/day, and the value of Electroencephalogram S/F in forehead, central, top, temporal, and occipital region in the PE group were all significantly higher than those in the no-PE group (*P* < 0.05) (Table 2).

### 3.3. Establishment of the Epilepsy after Encephalitis Predictive Model

The results of univariate logistic regression analysis showed that there were significant differences in the level of hemoglobin and globulin, the proportion of patients with fever or epilepsy frequency ≥10/day, and the value of electroencephalogram S/F in forehead, temporal, and occipital region between the PE group and no-PE group (Table 3). According to the results of univariate logistic regression analysis, we extracted the baseline characteristics of 255 patients with encephalitis, including hemoglobin and globulin, fever (no = 0, yes = 1), epilepsy frequency ≥10/day (no = 0, yes = 1), and the value of electroencephalogram S/F in the forehead, temporary and occipital regions, and analyzed whether the above factors affected the occurrence of epilepsy after encephalitis through multiple factor regression analysis. As shown, hemoglobin (OR = 0.968, 95% CI = 0.951–0.958), epilepsy frequency (OR = 0.968, 95% CI = 0.951–0.958), and ECG slow wave/fast wave frequency (S/F) in the occipital region were independent risk factors for PE (*P* < 0.05) (Table 4). Therefore, the corresponding predictive model was constructed based on the results of univariate and multiple logistic regression analysis. The model formula was as follows (hemoglobin is in g/L, epilepsy frequency ≥10/day = EF) : Model = −0.031 × Hemoglobin −2.113 × EF + 7.836 × Occipital region S/F + 1.595.

### 3.4. Evaluation of the Epilepsy after Encephalitis Predictive Model

Using the established model to calculate the model value of each encephalitis patient, we found that the model value of no-PE patients was significantly lower than that in PE patients in training set, validation set, and all patients (*P* < 0.05) (Figure 1). In addition, we also analyzed the predictive value of the model for PE and found that the area under the ROC curve (AUC) of the model for the diagnosis of PE in the training set and the validation set was 0.835 and 0.712, respectively (Figure 2). At the same time, the best cutoff value, sensitivity, and specificity value of the model were calculated based on ROC analysis (Table 5).

## 4. Discussion

Epilepsy is a clinical syndrome caused by the abnormal firing of highly synchronized neurons in the brain due to multiple causes. In China, the annual incidence of epilepsy is about 23/100,000, with more than 9 million epilepsy patients and 650,000–700,000 new epilepsy patients every year [18, 19]. The causes of epilepsy are complex, and epilepsy caused by structural damage or dysfunction of the central nervous system is called secondary epilepsy. Encephalitis is one of the common causes of secondary epilepsy, and 2.7% to 27.0% of patients with secondary epilepsy are associated with central nervous system infection and are easy to develop into refractory epilepsy [20, 21]. In this study, 46 of the 255 children with encephalitis were diagnosed with postencephalitis epilepsy; that is, the incidence was 18.04%, which is consistent with the previously reported incidence.

At present, the time definition of epilepsy after encephalitis is inconsistent in domestic and foreign studies. Annegers et al. retrospectively analyzed 714 adult patients with postencephalitis epilepsy and defined the acute phase within 2 weeks after the onset of encephalitis, and if the patient still had seizures after 2 weeks, it developed into postencephalitis epilepsy [22]. Wang-TSO et al. collected the case data of 330 pediatric encephalitis patients who had more than 2 seizures per month after applying more than 2 antiepileptic drugs as the screening criteria for postencephalitis epilepsy [23]. Tarun et al. defined postencephalitis epilepsy as seizures occuring more than 12 months after the acute phase of encephalitis with antiepileptic drugs [10]. Given that the damage to the central nervous system from encephalitis cannot be repaired in the short term and most children still require medical treatment for some time after encephalitis is discharged [24, 25]. Therefore, we defined epilepsy in children with encephalitis one year after hospital discharge as PE in this study.

In different studies on the influencing factors of epilepsy after encephalitis, different results have been obtained due to different types of patients and sample sizes, so the influencing factors of PE are still controversial [10, 11]. Singh et al. showed that interictal EEG abnormalities did not affect the development of PE, while seizure frequency and head MRI abnormalities in the acute phase of encephalitis were independent influencing factors affecting PE [10]. Liu et al. found that the influencing factors of PE after discharge from patients with anti-N-methyl-D-aspartate receptor encephalitis and viral encephalitis included seizures in the acute phase of encephalitis, status epilepticus, and admission to the ICU [11]. In children, seizure frequency, seizure type, impaired consciousness, and abnormal head neuroimaging are found to be risk factors for the development of PE [23, 26]. Herein, univariate and multiple logistic regression analysis showed that hemoglobin, epilepsy frequency, and ECG slow wave/fast wave frequency in the occipital region were independent influencing factors for PE.

Hemoglobin is a protein responsible for carrying oxygen in the human body. To our best efforts, no studies on hemoglobin in patients with PE have been reported, but there are many studies on hemoglobin and central nervous system injury. Previous studies found that hemoglobin not only changes when the human body is invaded by pathogens [27, 28], but also induces microglial inflammation [29, 30], causes oxidative damage, and causes the death of neurons [31, 32]. At the same time, hemoglobin was considered a strong predictor of clinical outcomes in patients with bacterial or viral infections [33, 34].

The frequency of epileptic seizures in the acute stage of encephalitis has been found by many studies to be an independent influencing factor of PE [10, 11], the same as in this study. The electrophysiological basis that causes epilepsy is the abnormal firing of neurons in the brain. After the acute phase of encephalitis, neurons in or near encephalitis lesions appear necrosis, deletion, structural disorders and malformations, blood supply disorders, biochemical metabolism disorders, less *γ*-aminobutyric acid synthesis, cell membrane proton pump imbalance, potassium outflow, calcium influx, and other pathological changes, in addition to continuous depolarization of neuronal cell membranes, which can also lead to abnormal firing of neurons, namely, secondary epilepsy [35, 36]. On the other hand, in the acute phase of encephalitis, each seizure increases the risk of damage to the central nervous system, neuronal excitotoxicity, and electrolyte imbalance, causing permanent nerve damage [37, 38]. EEG abnormalities have been linked to epilepsy in many studies [39, 40]. In view of the abnormal EEG in children with encephalitis, the main manifestation is the increase of slow waves, and the more severe the encephalitis, the greater the probability of high-amplitude slow waves [39, 40], so we included ECG slow wave/fast wave frequency in the analysis.

Based on the results of univariate and multivariate regression analysis, we established a model for predicting PE, and the ROC curve showed that the sensitivity and specificity of the model in predicting PE in children with encephalitis were high. A previous study has established a prediction model for epilepsy after Japanese encephalitis, ln (p/1p) = −3.533 + 1.103 × (seizures number > 5) + 1.366 × (status epilepticus) + 3.113 × (Coma) [41]. The sensitivity and specificity of this model in predicting epilepsy after encephalitis are 85.5% and 80.6%, respectively, which are lower than those in our study. In addition, some limitations of this study must be overstated: as a single center study, this study included a low sample size and had regional restrictions.

## Figures and Tables

**Figure 1:** Model value in encephalitis patients of training set, validation set and all patients. PE, postencephalitic epilepsy; no-PE, no postencephalitic epilepsy.

**Figure 2:** ROC curve regarding predictive value of model for epilepsy after encephalitis.

**Table 1:** Baseline characteristics of encephalitis patients in training set and validation set.

Variables	Training set (*n* = 184)	Validation set (*n* = 71)	t/*χ*2	*P*
Age (years)	7.78 ± 1.36	8.06 ± 1.62	1.407	0.161
Male (*n* (%))	129 (70.11)	55 (77.46)	1.380	0.240
WBC (x 10^9^/L)	9.23 ± 3.37	7.89 ± 2.65	1.614	0.108
NLR	6.06 ± 1.26	5.78 ± 1.57	0.331	0.741
Hemoglobin (g/L)	102.92 ± 24.53	104.39 ± 25.72	0.423	0.673
Platelet count (x 10^9^/L)	78.40 ± 61.35	78.06 ± 47.02	0.042	0.966
Albumin (g/L)	29.19 ± 6.33	28.78 ± 6.10	0.465	0.642
Globulin (g/L)	31.30 ± 6.81	31.88 ± 6.18	0.627	0.531
Epilepsy = first symptom (*n* (%))	54 (29.35)	19 (26.76)	0.168	0.682
Fever (*n* (%))	101 (54.89)	36 (50.70)	1.428	0.232
Consciousness disorder (*n* (%))	47 (25.54)	18 (25.35)	0.001	0.975
Partial seizure (*n* (%))	144 (78.26)	55 (77.46)	0.019	0.891
Epilepsy frequency ≥10/day (*n* (%))	26 (14.13)	11 (15.49)	0.077	0.782
MRI : Intracranial inflammation (*n* (%))	109 (59.24)	45 (63.38)	0.367	0.544

*Electroencephalogram slow wave/fast wave frequency*				
Forehead region	0.50 ± 0.20	0.48 ± 0.22	0.792	0.429
Central region	0.40 ± 0.20	0.39 ± 0.21	0.168	0.867
Top region	0.44 ± 0.15	0.45 ± 0.17	0.402	0.688
Temporal region	0.35 ± 0.12	0.38 ± 0.18	1.561	0.120
Occipital region	0.35 ± 0.13	0.35 ± 0.15	0.363	0.717

*Note.* WBC, white blood cell count; NLR, neutrophil to lymphocyte ratio.

**Table 2:** Baseline characteristics of encephalitis patients with or without postencephalitic epilepsy.

Variables	PE (*n* = 46)	No-PE (*n* = 209)	t/*χ*2	*P*
Age (years)	8.15 ± 1.62	7.80 ± 1.40	1.503	0.134
Male (*n* (%))	30 (65.22)	154 (73.68)	1.345	0.246
WBC (x 10^9^/L)	8.45 ± 3.02	9.05 ± 3.14	0.621	0.535
NLR	6.13 ± 2.09	5.95 ± 2.23	0.195	0.845
Hemoglobin (g/L)	88.28 ± 25.62	106.65 ± 23.45	4.728	<0.001
Platelet count (x 10^9^/L)	80.85 ± 56.11	7.74 ± 58.08	0.330	0.741
Albumin (g/L)	29.14 ± 4.31	29.06 ± 6.62	0.076	0.940
Globulin (g/L)	29.94 ± 6.57	31.80 ± 6.62	1.727	0.085
Epilepsy = first symptom (*n* (%))	15 (32.61)	58 (27.75)	0.435	0.509
Fever (*n* (%))	34 (73.91)	103 (49.28)	9.200	0.002
Consciousness disorder (*n* (%))	11 (23.91)	54 (25.84)	0.074	0.786
Partial seizure (*n* (%))	31 (67.39)	168 (80.38)	3.713	0.054
Epilepsy frequency ≥10/day (*n* (%))	17 (36.96)	20 (9.57)	22.797	<0.001
MRI : Intracranial inflammation (*n* (%))	22 (47.83)	122 (58.37)	1.706	0.191

*Electroencephalogram slow wave/fast wave frequency (S/F)*				
Forehead region	0.54 ± 0.15	0.48 ± 0.21	2.211	0.028
Central region	0.45 ± 0.17	0.37 ± 0.20	2.566	0.011
Top region	0.48 ± 0.13	0.43 ± 0.15	2.182	0.030
Temporal region	0.39 ± 0.13	0.34 ± 0.11	2.897	0.004
Occipital region	0.38 ± 0.12	0.32 ± 0.08	3.798	<0.001

*Note.* WBC, white blood cell count; NLR, neutrophil to lymphocyte ratio; PE, postencephalitic epilepsy.

**Table 3:** Univariate logistic regression analysis of influencing factors of epilepsy after encephalitis in the training set.

Variables	Coefficient	*P*	OR	95% CI
Age	0.193	0.158	1.213	0.928–1.587
Male	0.409	0.300	1.505	0.695–3.261
WBC	−0.001	0.967	0.999	0.942–1.059
NLR	0.002	0.939	1.002	0.944–1.065
Hemoglobin	−0.033	<0.001	0.968	0.951–0.985
Platelet count	0.002	0.555	1.002	0.996–1.007
Albumin	0.023	0.421	1.024	0.967–1.084
Globulin	−0.081	0.017	0.922	0.863–0.986
Epilepsy = first symptom	−0.285	0.477	0.752	0.344–1.648
Fever	−0.713	0.044	0.490	0.224–1.072
Consciousness disorder	−0.011	0.979	0.989	0.426–2.297
Partial seizure	−0.640	0.126	1.897	0.835–4.310
Epilepsy frequency ≥10/day	−1.616	<0.001	0.199	0.082–0.483
MRI : Intracranial inflammation	−0.660	0.107	0.517	0.232–1.152
Forehead region S/F	2.034	0.036	7.647	1.138–51.377
Central region S/F	1.424	0.116	4.155	0.705–24.481
Top region S/F	1.927	0.116	6.868	0.621–76.009
Temporal region S/F	3.200	0.041	24.537	1.145–525.820
Occipital region S/F	8.051	<0.001	138.273	74.695–138152.527

*Note.* S/F, electroencephalogram slow wave/fast wave frequency.

**Table 4:** Multivariate logistic regression analysis of influencing factors of epilepsy after encephalitis in the training set.

Variables	Coefficient	*P*	OR	95% CI
Hemoglobin	−0.031	0.004	0.969	0.949–0.990
Globulin	−0.052	0.200	0.950	0.878–1.028
Fever	−0.070	0.888	0.932	0.353–2.466
Epilepsy frequency ≥10/days	−2.113	<0.001	0.121	0.039–0.370
Forehead region S/F	1.392	0.267	4.024	0.345-46.921
Temporal region S/F	−1.152	0.592	0.316	0.005-21.218
Occipital region S/F	7.836	<0.001	2530.147	36.366–176036.044
Constant	1.595	0.462	4.929	

*Note.* S/F, electroencephalogram slow wave/fast wave frequency.

**Table 5:** Predictive value of the model for epilepsy after encephalitis.

	AUC	*P*	Cutoff value	95% CI	Sensitivity(%)	Specificity(%)
Training set	0.835	<0.001	3.8424	0.745–0.925	79.30	82.60
Validation set	0.712	0.0261	4.4495	0.469–0.956	87.70	90.00

## Data Availability

The data used to support the findings of this study are available from the corresponding author upon reasonable request.
